RETRACTED

# Different Amyloid-β Self-Assemblies Have Distinct Effects on Intracellular Tau Aggregation

**DOI:** 10.3389/fnmol.2019.00268

**Published:** 2019-11-08

**Authors:** Woo Shik Shin, Jing Di, Kevin A. Murray, Chuanqi Sun, Binsen Li, Gal Bitan, Lin Jiang

**Affiliations:** ^1^Department of Neurology, David Geffen School of Medicine, University of California, Los Angeles, Los Angeles, CA, United States; ^2^Department of Chemistry and Biochemistry, UCLA-DOE Institute, University of California, Los Angeles, Los Angeles, CA, United States; ^3^Department of Biological Chemistry, UCLA-DOE Institute, University of California, Los Angeles, Los Angeles, CA, United States; ^4^Brain Research Institute, University of California, Los Angeles, Los Angeles, CA, United States; ^5^Molecular Biology Institute, University of California, Los Angeles, Los Angeles, CA, United States

**Keywords:** amyloid beta, tau, biosensor cell, oligomer, Alzheimer’s disease

## Abstract

Alzheimer’s disease (AD) pathology is characterized by the aggregation of beta-amyloid (Aβ) and tau in the form of amyloid plaques and neurofibrillary tangles in the brain. It has been found that a synergistic relationship between these two proteins may contribute to their roles in disease progression. However, how Aβ and tau interact has not been fully characterized. Here, we analyze how tau seeding or aggregation is influenced by different Aβ self-assemblies (fibrils and oligomers). Our cellular assays utilizing tau biosensor cells show that transduction of Aβ oligomers into the cells greatly enhances seeded tau aggregation in a concentration-dependent manner. In contrast, transduced Aβ fibrils slightly reduce tau seeding while untransduced Aβ fibrils promote it. We also observe that the transduction of α-synuclein fibrils, another amyloid protein, has no effect on tau seeding. The enhancement of tau seeding by Aβ oligomers was confirmed using tau fibril seeds derived from both recombinant tau and PS19 mouse brain extracts containing human tau. Our findings highlight the importance of considering the specific form and cellular location of Aβ self-assembly when studying the relationship between Aβ and tau in future AD therapeutic development.

## Introduction

The accumulation of amyloid plaques and neurofibrillary tangles in the brain are the two major hallmarks of Alzheimer’s disease (AD) and are composed of the aggregated proteins β-amyloid (Aβ) and tau, respectively. Misfolded Aβ can aggregate to form soluble oligomers and insoluble fibrils (Glabe, 2008; Verma et al., 2015; Chiti and Dobson, 2017). Several studies have shown that oligomeric and fibrillar species of Aβ contribute differently to disease progression (Dahlgren et al., 2002; Li et al., 2014; Breydo and Uversky, 2015). For instance, Aβ oligomers, rather than Aβ fibrils, have been shown to be cytotoxic to neurons and play a significant role in cell death (Dahlgren et al., 2002).

RETRACTED

Although the amyloid cascade hypothesis posits Aβ accumulation as the initiating toxic event in AD, as reviewed by Hardy and Higgins (1992), the aggregation of tau, the other amyloid protein associated with AD, has drawn increased attention recently (Jouanne et al., 2017). Studies of biomarkers from patients correlate neurodegeneration and clinical decline to tau deposition independent of Aβ accumulation (Tapiola et al., 2009; Rosenmann, 2012; Dickerson et al., 2013). When tau aggregates into insoluble fibrils, these fibrillar species can act as a seed to facilitate further conversion of tau monomers into the fibrillar form (Kfoury et al., 2012; Jackson et al., 2016; Fitzpatrick et al., 2017). Tau seeding has been correlated with the development of tau pathology in the brain (DeVos et al., 2018; Kaufman et al., 2018).

Here, we aim to study the linkage between Aβ self-assembly and tau seeding. Many studies have analyzed the linkage of Aβ and tau in the context of AD, as recently reviewed (Leinonen et al., 2010; Ittner and Gotz, 2011; Bloom, 2014; Thal and Fandrich, 2015). The synergistic interaction between Aβ and tau has been highlighted in both animal models and biomarker study in patients (Spires-Jones and Hyman, 2014; Bennett et al., 2017; Busche et al., 2019). The animal model study has shown the synergistic incensement of tau accumulation in the presence of Aβ in the cortex of young tau (P301L)-overexpressed mice (He et al., 2018; Vergara et al., 2019). Also, biomarker studies in patients suggest that the progression to dementia is driven by the interaction between Aβ and tau (Mulder et al., 2010; Dickerson et al., 2013; Pascoal et al., 2017). Furthermore, additional studies show that rather than just toxicity, Aβ can lead to other cellular responses related to the development of tau pathology, such as increased tau phosphorylation (Zheng et al., 2002; Sun et al., 2008; Ma et al., 2009). However, the molecular mechanism by which Aβ influences tau seeding and aggregation, specifically which aggregate species of Aβ contributes most to this process, is unknown.

To dissect the contributions different self-assemblies of Aβ have on tau seeding, a method for quantitatively studying tau seeding is needed. The HEK293T tau biosensor cell line developed by Diamond and co-workers is capable of monitoring and quantifying intracellular tau aggregation and seeding (Holmes et al., 2014; Furman et al., 2015). Expressing tau RD containing the disease-associated P301S substitution fused to either cyan or yellow fluorescent proteins (CFP/YFP), the biosensor cells produce a FRET signal upon aggregation of tau, which can be quantified using flow cytometry. In this study, we sought to explore how different Aβ assemblies might contribute to the process of tau seeding. We use the biosensor cells to measure the unique contributions of different assemblies of Aβ – freshly prepared, oligomeric, and fibrillar – on tau seeding.

RETRACTED

## Results

To determine the effects of different forms of amyloid beta self-assemblies on intracellular tau seeding, we first generated and characterized three forms of Aβ self-assemblies: freshly prepared, oligomeric, and fibrillar. Recombinant Aβ42 was expressed and purified as described previously (Jiang et al., 2013). After purification, Aβ was diluted in PBS (10 μM), yielding a sample composed of a single band and a mixture of several low molecular weight higher-order assemblies, as assessed by native PAGE (Supplementary Figure 1b). We term this sample “freshly prepared” Aβ. After quiescent incubation at 37°C for 18 h, the Aβ aggregated into spherical oligomers, as shown by electron microscopy (EM) (Figure 1B). After continued incubation for a total of 100 h, the Aβ formed long, unbranched amyloid fibrils. Aggregation was assessed by Thioflavin T (ThT) fluorescence (Supplementary Figure 1a), which indicates the presence of fibrillar Aβ.

**FIGURE 1:** Aggregate species (freshly prepared, oligomeric, fibrillar) of Aβ have distinct effects on tau seeding. **(A)** Schematic of HEK293T tau biosensor cell seeding assay. Cells are transduced with Aβ, followed by tau fibril seeds 24 h later. Aggregation of tau can be detected by the presence of a FRET signal. **(B)** EM images of Aβ self-assemblies (freshly prepared, oligomeric, and fibrillar) used in seeding experiments. **(C)** Fluorescent microscope images of seeded biosensor cells taken in the green channel (ex. 488 nm, em. 520 nm). Background fluorescence (control, left panel) is diffuse non-aggregated YFP-tau. With the addition of tau seeds, the endogenous tau aggregates into small discrete fluorescent puncta. Before the addition of tau fibril seeds, cells are pretreated with different self-assembly forms of Aβ. **(D)** Flow cytometry quantification shows that increasing pretreatment concentrations of Aβ oligomers enhance intracellular tau aggregation seeded by tau fibrils (50 nM), while freshly prepared Aβ has little effect. Aβ fibrils show slight inhibition of tau seeding. Seeding is measured by Integrated FRET Density (IFD). **(E)** Tau seeding in biosensor cells seeded with increasing concentrations of tau fibrils and pretreated with different forms of Aβ. The data are presented as mean ± SD (*n* = 9).

RETRACTED

To measure the effects of Aβ aggregates on intracellular tau aggregation, we utilized tau HEK293T biosensor cells, which express the repeat domain of tau (tau RD) with the P301S mutation, fused with either yellow fluorescent protein (YFP) or cyan fluorescent protein (CFP) (Holmes et al., 2014). Upon aggregation of tau within the biosensor cell, the YFP and CFP form a FRET pair, allowing for spectroscopic quantification of the number of aggregates that form (Figure 1A). Cells were initially transduced with different Aβ species (freshly prepared, oligomeric, and fibrillar; Figure 1B) using lipofectamine, followed by transduction of fibrillar tau RD seeds 24 h later. After an additional 24 h, cells were imaged by fluorescent microscopy, and they were then harvested for analysis by flow cytometry 24 h after imaging. Without transduction of any tau seeds, the biosensor cells show a diffuse fluorescent signal, indicating background expression of non-aggregated endogenous tau. Images of the biosensor cells seeded with tau RD (10 nM) show intracellular tau aggregates in the form of bright fluorescent puncta (Figure 1C). The number of visible puncta greatly increases with a rising concentration of Aβ oligomers, but a much smaller effect is observed with the freshly prepared Aβ. Aβ fibrils appear to have a slight inhibitory effect on tau seeding. These seeding effects were quantified by FRET-based flow cytometry, which measures intracellular tau aggregation using integrated FRET density (IFD, FRET intensity multiplied by the percentage of FRET + cells). The flow data show that the enhancement of tau seeding by Aβ oligomers is dose-dependent, while the effects of freshly prepared and fibrillar Aβ are much less obvious (Figure 1D). We then further characterized these different effects by varying the amount of tau fibril seeds used in the seeding assay. Cells were pretreated with the three different Aβ species (100 nM) and increasing tau fibril seed concentrations (1–200 nM). The effects of each Aβ species on tau seeding are much more pronounced with higher tau seed concentrations: Aβ oligomers enhance seeding, Aβ fibrils have an inhibitory effect, and freshly prepared Aβ has little effect (Figure 1E). We also performed a seeding experiment using Aβ treatment without transfection reagent lipofectamine (Supplementary Figure 3). When different concentrations of Aβ assemblies are added to culture media without lipofectamine, Aβ fibrils and freshly prepared Aβ promote tau seeding in a dose-dependent manner, and Aβ oligomers show stronger promotion.

We further analyzed the effects of Aβ oligomers on the promotion of tau seeding with a broader range of tau fibril seed concentrations (Figure 2). Tau biosensor cells seeded with increasing concentrations of tau RD display increased tau aggregation as quantified by flow cytometry (Figure 2A) and confirmed by fluorescent imaging (Figure 2B). The addition of Aβ oligomers at 200 nM halves the amount of tau fibril seeds needed to seed tau biosensor cells (EC_50_: 60 nM) as compared to cells with no pretreatment (EC_50_: 125 nM). We then sought to determine if the effects of Aβ oligomers on tau seeding are specific to Aβ or if other amyloid proteins might lead to similar seeding enhancement. Pretreatment of biosensor cells with α-synuclein fibrils (500 nM) showed no effect on tau seeded (EC_50_: 120 nM), comparable to cells with no pretreatment. This indicates that tau seeding is promoted by Aβ oligomers but not α-synuclein.

RETRACTED

**FIGURE 2:** Tau seeding is specifically enhanced by Aβ, not α-synuclein. **(A)** Tau seeding of biosensor cells pretreated with transduced α-synuclein fibrils or Aβ oligomers as measured by Integrated FRET Density (IFD). **(B)** Representative fluorescent images of treated tau biosensor cells. The data are presented as mean ± SD (*n* = 9).

The generation of recombinant tau fibril seeds is traditionally done in the presence of aggregation inducers such as heparin. In our seeding experiments, fibril seeds were generated under high protein concentration in the absence of any aggregation inducer, as it has been reported that such molecules may have complicated effects on tau aggregation and seeding. We aimed to determine whether the promotion of tau seeding by Aβ oligomers is dependent on heparin. To test this, we generated tau fibril seeds grown in the presence of heparin and compared tau seeding with and without heparin (Supplementary Figure 2). At low concentrations of tau seed, the fibrils grown with heparin increase seeding relative to fibrils without heparin. However, at high concentrations, the seeding levels are similar. When cells are pretreated with Aβ oligomers, the promotion of tau seeding is still observed with and without heparin (Supplementary Figure 2c).

Following the observation that Aβ oligomers enhance biosensor cell seeding with recombinant tau RD, we then determined whether other forms of tau seeds lead to similar effects. Brain extract of transgenic PS19 mice, expressing full-length P301S human tau, was used as a tau seed. The seeds were extracted from the mouse brains using previously published methods (Jackson et al., 2016; Goedert and Spillantini, 2017). The concentration of human tau in the brain extracts was quantified using ELISA (see section “Materials and Methods”). Similar to recombinant tau RD, the mouse brain extract seeding was greatly enhanced by pretreatment with Aβ oligomers (Figure 3).

RETRACTED

**FIGURE 3:** Aβ promotes tau seeding with brain extract from mice expressing human full-length P301S tau. **(A)** Tau seeding of biosensor cells transduced with PS19 mouse brain extract as measured by Integrated FRET Density (IFD). The concentration of human tau in the brain extracts was quantified using ELISA. The data are presented as mean ± SD (*n* = 6). **(B)** Representative fluorescent images of treated tau biosensor cells.

## Discussion

The aggregation of amyloid beta follows the conversion of monomers into small soluble oligomers and then the eventual growth of fibrils. The different aggregate species that are generated in this aggregation process may have drastically different biological effects. Previous work has indicated that Aβ aggregates have different cytotoxicities and have unique contributions to AD progression (Dahlgren et al., 2002; Heo et al., 2007; Li et al., 2014). Our experiments quantitatively study the effects of different Aβ aggregates on tau seeding, another important contributor to AD pathology. We demonstrate that internalized Aβ fibrils and oligomers are opposite in their effects on tau seeding. Aβ oligomers show promotion of tau seeding and fibrils show a reduction, while freshly prepared Aβ had no obvious effects on seeding. It is possible that the observed difference in tau seeding between Aβ fibril- and oligomer-treated cells is a result of the potentially lower transfection efficiency of Aβ fibrils compared to oligomers due to their larger size. We observe that the addition of Aβ fibrils decreases the amount of tau seeding not only relative to Aβ oligomers but also relative to cells in which no Aβ was added. If this decrease in tau seeding caused by Aβ fibrils is only due to lower transfection efficiency, then we expect that the tau seeding with transfected Aβ fibrils will be lower relative to with Aβ oligomers but greater or equal to the seeding in cells with no Aβ. However, we observe that the tau seeding with Aβ fibrils is lower than the levels in the cells with no Aβ, indicating that the effects are not just due to concentration and that the transfected Aβ fibrils have distinct effects on tau seeding compared to oligomers.

To further explore the contribution of transfection efficiency, we performed control seeding experiments without the use of transfection reagent lipofectamine. Without the use of lipofectamine to transfect the Aβ species into the cell, Aβ oligomers and fibrils both enhance tau seeding (Supplementary Figure 3). These findings agree with recent publications that have focused on cross-seeding between Aβ and tau fibrils, in which aggregated Aβ promotes the formation of tau aggregates (Stancu et al., 2014; Bennett et al., 2017; He et al., 2018). Our *in vitro* cellular experiments show that transfected Aβ fibrils inhibit tau seeding, while non-transfected Aβ fibrils enhance it. The results of this study performed in a model cell system suggest that intracellular and extracellular Aβ fibrils have opposite effects on intracellular tau aggregation. This also highlights the fact that the impact of Aβ on tau seeding is dependent on the location of its aggregate form. This may have broader implications for the nature of AD disease progression, in that the seeding of tau aggregation and subsequent development of tau pathology is dictated by which aggregate species of Aβ are present and where they are located. This highlights the importance of considering the location and type of amyloid species when developing assays to design and screen therapeutics targeting Aβ and tau pathology.

RETRACTED

Our cell culture model utilizes tau biosensor cells expressing tau RD fused with CFP/YFP. The repeat domain has been shown to contain the amyloid fibril core of tau, as supported by the recently published tau paired-helical filament structure from patient brains (Fitzpatrick et al., 2017; Falcon et al., 2018). A potential limitation to this cell culture model could be present if segments of tau outside of the RD (i.e., use of full-length tau) contribute to seeding and fibrillization. Nevertheless, these biosensor cells are a useful tool to assess tau seeding *in vitro*, as they can be seeded with tau fibrils from various *in vitro* and *in vivo* sources, both truncated and full-length (Sanders et al., 2014; Kaufman et al., 2016).

Our study partially relies on the use of recombinant tau fibrils to assess the role of Aβ on tau aggregation. Traditionally, *in vitro*-generated tau fibrils are grown in the presence of heparin, which is known to induce aggregation (Friedhoff et al., 1998; King et al., 1999). Due to the complicated role of heparin on the tau aggregation process, the application of tau seeds in the presence of heparin may introduce confounding effects. Thus, we attempted to explore the use of a heparin-free system in our seeding experiments. In this study, we generated the recombinant tau fibrils without the use of heparin, relying on relatively high concentrations of tau monomer to facilitate aggregation. Growth of tau fibrils without heparin displayed similar aggregation kinetics as monitored by ThT fluorescence (Supplementary Figure 2), and EM imaging shows long unbranched fibrils similar in morphology to published images of tau RD with heparin (Nizynski et al., 2018). Comparison of biosensor cells seeded with tau fibrils grown in the presence or absence of heparin show that both fibril preparations can seed the cells but that the seeding capacities of each preparation are different. It is possible that these observed differences in seeding are influenced by the heparin. Using fibrils grown without heparin ensures that the seeding effects measured in this study come directly from tau fibrils. These findings demonstrate that it is practical to use recombinant fibrils grown without heparin in future seeding and aggregation studies, avoiding any potential complications with the use of aggregation inducers.

RETRACTED

## Materials and Methods

### Aβ Expression and Purification

Aβ (1–42) was expressed and purified as described previously (Jiang et al., 2013; Cao et al., 2018). The fusion protein of Aβ(1–42) with maltose-binding protein (MBP – Aβ42) was expressed using *Escherichia coli* BL21 plyS (DE3) cells and then purified using a HisTrap HP column (GE healthcare). After overnight cleavage by TEV protease, the uncleaved protein and TEV were removed using Ni^2+^ affinity chromatography. The Aβ(1–42) in the flow-through was purified by RP-HPLC and lyophilized. The homogeneity of the Aβ sample was ensured by dissolving the lyophilized powder in 60 mM NaOH and then fractionating it by SEC (GE, Superdex 200 Increase) in 20 mM NaOH to eliminate pre-formed Aβ aggregates. The final concentration was determined by a BCA assay, and the stock was stored at −80°C.

### Tau Expression and Purification

Human tau RD (residues 244–372) was expressed and purified as described previously (Seidler et al., 2018). Briefly, BL21 (DE3 GOLD) competent *E. coli* cells and a pNG2 vector were used for the expression of tau RD. After sonication, cell lysates were boiled for 20 min and centrifuged to remove all insoluble proteins. The remaining soluble protein was purified using a HighTrap SP ion-exchange column (GE Healthcare), and fractions were analyzed by SDS-PAGE/Coomassie blue staining. Enriched fractions were further purified using a HiLoad 16/600 Superdex 75 SEC column (GE Healthcare). Purified tau was concentrated to 50–100 mg/ml and stored at −80°C.

### Thioflavin T Kinetics of Aβ Self-Assembly

Before the ThT kinetics assay, freshly SEC-fractionated Aβ was mixed with 60 mM HCl to neutralize the NaOH in the stock solution. The Aβ sample was then diluted in PBS to a final concentration of 10 and 30 μM ThT (CalbioChem) was added. The reaction mixture was filtered through a 0.2-μm filter and immediately placed in a Corning 96-well Non-binding plate (black, non-binding surface microplate) at 100 μl per well. The ThT fluorescence signal was measured every 5 min in quiescent conditions using a Fluostar Omega plate reader (BMG Labtech, Offenburg, Germany) with excitation and emission wavelengths of 440 and 490 nm, respectively, at 37°C.

RETRACTED

### Thioflavin T Kinetics of Tau Aggregation With and Without Heparin

Freshly purified tau RD was diluted in PBS containing 2 mM DTT and 40 μM ThT to a final concentration of 200 μM in the absence of any aggregation inducers (i.e., heparin). For tau with heparin, sample tau RD (final concentration: 20 μM) was diluted in PBS containing 2 mM DTT, 40 μM ThT, and heparin (0.5 mg/ml). The reaction mixture was split into 3–4 replicates and placed in 96-well plates (Corning 3881) at 100-μL well volumes. ThT fluorescence intensity was measured every 15 min with double orbital shaking at 37°C in the same plate reader until a plateau was reached.

### Measurement of Tau Seeding Using HEK293T Biosensor Cells

Tau RD P301S FRET Biosensor (ATCC CRL-3275) cells were cultured and analyzed as described previously (Holmes et al., 2014; Furman et al., 2015). Briefly, HEK293T cells were plated on collagen-coated flat 96-well plates at a density of 2.5 × 10^4^ cells/well in 200 μl of culture medium and incubated at 37°C in 5% CO_2_. After 24 h, the cells were transduced with different self-assembly states of Aβ or sonicated α-synuclein fibrils. The preparation of recombinant α-synuclein fibrils was performed as described previously (Li et al., 2018). For protein transduction, Aβ or α-synuclein was first diluted into Opti-MEM media (GIBCO) at a 1:20 ratio, and Lipofectamine^TM^ 2000 (Thermo Fisher Scientific) was also diluted in Opti-MEM at a 1:20 ratio. The protein and lipofectamine dilutions were then mixed at equal volumes and incubated for 15 min before application to cells. Tau fibril seeds were transduced into the cells 24 h after Aβ/α-syn transduction. Tau fibrils (tau RD and mouse brain extract) were first diluted with Opti-MEM (1:20 ratio) and sonicated for 10 min in an ultrasonic water bath then mixed with a 1:20 lipofectamine dilution and incubated for 15 min. Tau aggregation in the biosensor cells was visualized by fluorescence microscopy 24 h after tau fibril seed transduction using the green channel (ex: 485 nm; em: 520 nm). The cells were harvested 24 h after imaging after extensive washing and treatment with trypsin. The harvested cells were prepared in 200 μl of chilled buffer (HBSS, 1% FBS, 1 mM EDTA) and then stored at 4°C until they were analyzed by FRET-based flow cytometry.

### Flow Cytometry and Data Analysis of Tau Seeding

Intracellular protein aggregation of tau was quantified using FRET-based flow cytometry with an adapted protocol (Furman et al., 2015) using a Digital Analyzers LSRII (IMED) flow cytometer. The fluorescence intensities of the FRET signal were measured (ex: 405 nm; em: 525/50 nm), and CFP-fusion proteins (ex: 405 nm; em: 405/50 nm) and YFP-fusion proteins (ex: 488 nm; em: 525/50 nm) alone were measured for background subtraction. For each experiment, FRET signals of 20,000 cells per replicate were analyzed. FRET gating was introduced to exclude all FRET-negative cells and include the FRET-positive cells. Integrated FRET density (IFD), defined as the percentage of FRET-positive cells multiplied by the median fluorescence intensity of FRET-positive cells, was calculated for all analyses.

RETRACTED

### Electron Microscopy

Aliquots of 3∼5 μl from aggregation reactions were taken at different time points and applied to carbon-coated 400-mesh Formvar grids (Electron Microscopy Science) that had been glow-discharged using a Pelco Easy-Glow unit immediately before sample application. The samples were stained with 2% uranyl acetate and analyzed using a JEOL JEM1200-EX transmission electron microscope.

### Animals

Animal care was conducted in compliance with the United States Public Health Service Guide for the Care and Use of Laboratory Animals, and the procedures were approved by the Institutional Animal Care and Use Committee at the University of California, Los Angeles. Eight-month-old P301S (PS19) transgenic mice on (C57BL/6 × C3H) F1 background mice were used for the study.

### Preparation of Mouse Brain Extracts

Eight-month-old PS19 mice and age-matched WT mice were deeply anesthetized with isoflurane (0.5–1.5 vol% in oxygen) and sacrificed by decapitation. Brains were dissected and suspended in 10% (w/v) ice-cold TBS containing protease and phosphatase inhibitors cocktail (ThermoFisher). The tissue was homogenized at 4°C using a probe sonicator (Omni Sonic Ruptor 250) at 30% power using 25 pulses. Lysates were centrifuged at 21,000 × g for 15 min to remove cell debris. Supernatants were aliquoted and stored at −80°C. Tau concentration was quantified using an anti-tau ELISA kit (Invitrogen, cat# KHB0041) according to the manufacturer’s instructions.

### Statistical Analyses

All graphs were generated using Prism software ver. 7.0 (San Diego, CA, United States). The EC_50_ values and plots were determined by fitting the data to a sigmoidal dose-response curve. All FRET quantifications were conducted for a minimum of three independent experiments, with at least three replicates in each experimental condition.

## Data Availability Statement

All datasets generated for this study are included in the article/Supplementary Material.

RETRACTED

## Ethics Statement

Animal care was conducted in compliance with the United States Public Health Service Guide for the Care and Use of Laboratory Animals, and the procedures were approved by the Institutional Animal Care and Use Committee at the University of California, Los Angeles. Eight-month-old P301S (PS19) transgenic mice on (C57BL/6 × C3H) F1 background mice were used for the study.

## Author Contributions

LJ designed and supervised the research. WS performed cellular seeding, flow cytometry, ELISA experiments, florescence microscope imaging, and analyzed the data. JD and GB prepared mouse brain extracts. CS and BL purified Aβ protein. WS purified tau protein. WS, KM, CS, and BL characterized the self-assembly of Aβ and tau protein. WS, KM, and LJ wrote the manuscript with the input from all authors. All authors read and approved the final manuscript.

## Conflict of Interest

The authors declare that the research was conducted in the absence of any commercial or financial relationships that could be construed as a potential conflict of interest.
